This article has been retracted.

# Development and Evaluation of Fluorescence Immunochromatography for Rapid and Sensitive Detection of Thermophilic *Campylobacter*

**DOI:** 10.14252/foodsafetyfscj.D-21-00006

**Published:** 2021-09-24

**Authors:** Hiroshi Asakura, Junko Sakata, Yoshimasa Sasaki, Kentaro Kawatsu

**Affiliations:** 1 Division of Biomedical Food Research, National Institute of Health Sciences, 3-25-26 Tonomachi,Kawasaki-ku, Kawasaki 210-9501, Japan.; 2 Bacteriology Section, Osaka Institute of Public Health, 1-3-69 Nakamichi, Higashinari-ku, Osaka 537-0025, Japan.

**Keywords:** *Campylobacter*, fluorescence immunochromatography (FIC), poultry slaughter, process hygiene

## Abstract

*Campylobacter jejuni* (*C. jejuni*) and *Campylobacter coli* (*C. coli*) are leading causes of foodborne gastroenteritis in Japan. Epidemiological surveillance has provided evidence that poultry meat is one of the main reservoirs for human campylobacteriosis, and therefore, improvement in process hygiene at slaughter is required to reduce the number of human infections. This study thus aimed to develop fluorescent immunochromatography strips for rapid and sensitive detection of thermophilic *Campylobacter* on poultry carcasses at slaughter. To establish the required detection levels, we first determined the numbers of *C. jejuni* and *C. coli* on poultry carcasses at one large-scale poultry slaughterhouse in Japan, resulting in the detection of *Campylobacter* at 1.97 ± 0.24 log CFU/25 g of neck skin during the post-chilling process by using ISO 10272-2:2017. Our developed *Campylobacter* fluorescence immunochromatography (FIC) assay exhibited a 50% limit of detection of 3.51 log CFU or 4.34 log CFU for *C. jejuni* NCTC 11168 or *C. coli* JCM 2529, respectively. Inclusive and exclusive tests resulted in good agreement. The practical usefulness of this test toward poultry carcasses should be evaluated in future studies, perhaps concentration of the target microorganisms prior to the testing might be helpful to further enhance sensitivity. Nevertheless, our data suggest the potential of FIC for rapid and sensitive detection of thermophilic *Campylobacter* for monitoring the process hygiene of poultry carcasses at slaughter.

## Introduction

*Campylobacter jejuni (C. jejui) and Campylobacter coli (C. coli)* are the leading causes of foodborne gastroenteritis worldwide, particularly in developed countries^1^^)^. Similar to in Western countries^2^^,^^3^^)^, poultry meat and its products are recognized as some of the major reservoirs for human campylobacteriosis in Japan^4^^)^. Thus, it is necessary to monitor and improve the hygienic status of poultry processing at slaughter to reduce human campylobacteriosis.

In this regard, the European Food Safety Agency (EFSA) performed a baseline survey and concluded that broiler carcasses were contaminated at an average of 75.8%, with significant variations between member states and slaughterhouses^5^^)^. The EFSA also estimated that the public health risk from the consumption of broiler meat could be reduced by more than 50% if the poultry carcasses complied with a limit of 3.0 log CFU/g of neck skin^6^^)^. Based on this evidence, the Food Safety Authority of Ireland (FSAI) amended Regulation (EC) No 2073/2005 to newly set a process hygiene criterion for *Campylobacter* at slaughterhouses and, in January 2018, started to monitor the bacterial burden^7^^)^.

To monitor the bacterial contamination levels on poultry carcasses, the FSAI recommended using ISO 10272-2, an international standard method to quantitatively detect the numbers of thermophilic *Campylobacter*, which is mainly composed of direct plating onto selective agar and subsequent confirmation testing^8^^)^. However, such a standard method is time-consuming and requires technical capability to obtain accurate results mainly due to the bacterial characteristics, such as their microaerophilic nature^1^^)^. In the slaughter field, easy-to-use and rapid technologies are expected to allow continuous monitoring. However, such an alternative method should putatively detect approximately 3.0 log CFU of *C. jejuni* and *C. coli* in order to achieve a 50% reduction in public health risk, as recommended by the FSAI.

To date, several chronometric immunochromatography strips have been developed, most of which show a sensitivity of more than 5.0 log CFU of *Listeria monocytogenes*^9^^)^ and *Salmonella* spp.^10^^)^. For *Campylobacter*, a previous study also developed chronometric immunochromatography for its rapid detection from human clinical specimens in combination with preenrichment culture; however, the detection limits of this method ranged from 4.3 to 5.9 log CFU/mL for *C. jejuni* and 5.1 to 6.7 log CFU/mL for *C. coli*^11^^)^. Further study showed that a chronometric immunochromatography kit showed sensitivity at 8.0 log CFU/g from chicken feces^12^^)^. These are likely to be insufficient for bacterial monitoring at slaughter, as mentioned above.

A recent advancement in fluorescent silica nanoparticle technology enables us to develop sensitive assay systems for the detection of a series of target molecules^13^^)^. Indeed, fluorescent silica nanoparticles have been used for the development of rapid detection and/or diagnostic tools for clinical specimens for *Acanthamoeba keratitis*^14^^)^, *Salmonella*^15^^)^, *Staphylococcus aureus*^16^^)^, and *Escherichia coli* O157^17^^)^. As fluorescent silica nanoparticles show binding affinity to immunoglobulins^18^^)^, the particles might be utilized for construction of a sensitive immunochromatography system for thermophilic *Campylobacter*.

Given this background, we aimed to develop a fluorescent immunochromatography (FIC) assay for rapid and sensitive detection of *Campylobacter*, and its performance was evaluated by estimating the 50% limit of detection (LOD_50%_) as well as inclusive/exclusive testing as qualitative testing method.

## Materials and Methods

### Samples

Neck skins were taken from poultry carcasses at post-defeathering, post-evisceration and post-chilling processes at one large-scale poultry slaughterhouse in Japan, which processes approximately 75,000 broilers per day on average. The skins from five birds were pooled to obtain 25 g (designated as a skin sample), and 15 samples were prepared at three processing points collected from the same lot on the same day.

### Quantitative Detection of *Campylobacter* from Poultry

Thermophilic *Campylobacter* was quantitatively detected from poultry neck skin samples essentially according to ISO 10272-2:2017^8^^)^. Briefly, after homogenization with 225 mL of buffered peptone water (Oxoid, Hampshire, UK), a total of 1 mL of the homogenates and serial dilutions were spread on modified charcoal-cefoperazone-deoxycholate agar plates (Oxoid), followed by microaerophilic incubation at 41.5 °C for 48 h using an AnaeroPack-Microaero (Mitsubishi Gas Chemicals, Tokyo, Japan). Per sample, five suspected colonies grown on the plates were subjected to PCR-based identification using *C. jejuni*- and *C. coli*-specific primers, as previously described^19^^)^.

### Development of a *Campylobacter* fluorescence Immunochromatography (FIC) assay as Qualitative Detection Method

Membrane-based lateral flow immunochromatographic strips with fluorescent nanoparticles were constructed by Furukawa Advanced Engineering, Japan (Chiba, Japan). In brief, a mouse anti-*Campylobacter* monoclonal antibody (MAb)^11^^)^ was conjugated with fluorescent silica nanoparticles (Quartz Dot^®^; Furukawa Advanced Engineering) as previously described^18^^)^. The prepared MAb-fluorescent silica nanoparticle conjugates were suspended in 1.0 mL of 50 mM Tris-HCl/150 mM NaCl/1% bovine serum albumin/20% glycerol and then freeze-dried before storage at -30 °C until use. To construct a test strip, an absorbent pad (Millipore, Bedford, MA, USA) was attached to a laminated membrane card (Whatman FP, Cytiva, Marlborough, MA, USA) so that the pad slightly overlapped the membrane, and the assembly was then cut into strips consisting of the membrane (5 by 25 mm) with the absorbent pad (5 by 17 mm). One microliter aliquots of the MAb-Quartz Dot^®^ conjugates were deposited on the membrane, which was stored in the dark until use.

### Determination of the Specificity of the *Campylobacter* FIC Assay

For inclusive testing, a total of 55 bacterial strains, including 25 *C. jejuni*, 25 *C. coli*, and 5 *Campylobacter lari* (*C. lari*) strains, were subjected to the *Campylobacter* FIC assay. For exclusive testing, 5 *Campylobacter fetus*, 3 *Campylobacter upsaliensis*, 3 *Campylobacter hyointestinalis* strains and non-*Campylobacter* bacterial strains (10 *Escherichia coli*, 10 *Salmonella* spp., 10 *Arcobacter butzeleri*, 4 *Enterobacter* spp., 1 *Klebsiella aerogenes*, 1 *Shigella flexneri*, 5 *Pseudomonas* spp., and 5 *Helicobacter pylori* strains) were used. These bacterial strains were generally cultured in Mueller-Hinton broth (Becton Dickinson, Franklin lakes, NJ, USA), except for *H. pylori*, which was cultured in Brucella broth (Becton Dickinson) supplemented with horse serum (Thermo Fisher Scientific), then followed by washing twice with sterile phosphate-buffered saline (PBS). The bacterial pellets were resuspended in PBS to achieve approximately 8.0 to 8.3 log CFU/mL, and 50 μL aliquots of these suspensions (equivalent to approximately 6.7 to 7.0 log CFU) were then added to equal volumes of the B-PER II reagent (Thermo Fisher Scientific, Waltham, MA, USA). After homogenization in microtubes with zirconia beads (Zircoprep Mini, Nippon Genetics, Tokyo, Japan) on a Digital Disruptor Genie (Scientific Industries, Bohemia, NY, USA) at 2,850 rpm for 5 min, the homogenates were centrifuged at 10,000 x *g* at 4°C for 5 min. The resulting supernatants (crude extracts) were applied to the *Campylobacter* FIC assay strip. At 15 min post loading, the appearance of detectable bands for *Campylobacter* antigens was visually monitored by using a fluorescence hand scope (Furukawa Advanced Engineering). PBS alone was used as a negative control.

### Determination of the Sensitivity of the *Campylobacter* FIC Assay

The sensitivity of the *Campylobacter* FIC assay was examined using different numbers (a total of 6 inoculation levels) of *C. jejuni* NCTC 11168 and *C. coli* JCM 2529 cells grown on Mueller-Hinton agar (Becton Dickinson) at 41.5 °C for 24 h under a microaerobic atmosphere. Following two washes with PBS, a bacterial suspension (corresponding to 6.0 to 6.6 log CFU/50 µL) and serial 10-fold dilutions were prepared in PBS (Thermo Fisher Scientific), and 50 µL aliquots of each dilution were processed as mentioned above. Simultaneously, the cell suspensions were spread onto Mueller-Hinton agar to enumerate CFU. PBS alone was used as a negative control. This test was performed in 5 independent sets, and the LOD_50%_ was calculated accordingly^20^^)^.

## Results and Discussion

### Quantitative Detection of Thermophilic *Campylobacter* on Broiler Carcasses at Slaughter

We first examined the quantitative detection of thermophilic *Campylobacter* on broiler neck skin samples collected at three processing points in one poultry slaughterhouse according to ISO 10272-2:2017. Overall, all samples were positive for *Campylobacter*. At post-defeathering, *Campylobacter* was detected at levels ranging from 3.48 to 5.27 log CFU/sample (25 g) of neck skin (mean ± SD of 4.21 ± 0.78 log CFU/25 g) (Fig. 1). The bacterial counts were then increased after the evisceration process to 4.78 ± 0.46 log CFU/25 g on average (4.30 to 5.43 log CFU/25 g) (Fig. 1), suggesting the occurrence of cross-contamination of this pathogen on the carcass during evisceration. The carcasses at the post-chilling process thereafter exhibited decreased bacterial contamination levels at 1.97 ± 0.24 log CFU/25 g on average (1.70 to 2.30 log CFU/25 g) (Fig. 1), which indicated that the chilling process effectively reduced bacterial contamination. An interview of the slaughterhouse personnel confirmed that the chilling tank contained 30 ppm sodium hypochlorite at <5 °C for >30 min, which was set as the critical control point by the facility. As chilling and antimicrobial treatment have usually been combined in many processing plants to save energy and rapidly inhibit bacterial survival and growth by washing the carcasses with cold chlorinated water^21^^)^, our data indicated that the target facility maintained good manufacturing control during the chilling process. Nevertheless, the samples at the post-chilling process possessed approximately 2.0 log CFU/25 g *Campylobacter*, suggesting the further necessity to reduce the bacterial contamination; accordingly, quantitative microbial risk assessments have validated the effectiveness of interventions such as scalding and chilling during processing by reporting an average of 4.0 log reductions in *Campylobacter* concentrations from before processing to immediately after carcass chilling^22^^)^, but the current process examined herein did not satisfy such criteria. The facility is encouraged to confirm the adequacy of chemical antimicrobial interventions, as several more effective antimicrobials have been reported to date^23^^)^.

**Fig. 1.** Quantitative detection of thermophilic *Campylobacter* from poultry carcasses at slaughter. Neck skin samples were taken at the postdefeathering, postevisceration and postchilling processes. Means represent the bacterial numbers as log CFU/g.

### Specificity of the *Campylobacter* FIC Strip

The quantitative detection procedure of *Campylobacter* could provide useful information for risk management in the slaughter process, as well as evaluation of the efficiency of the adopted intervention^24^^)^. To perform continuous monitoring, practical approach with reduced costs and times for screening highly contaminated carcasses is seemingly expected. To address this issue, we developed an FIC assay for rapid and sensitive detection of thermophilic *Campylobacter*, which can obtain qualitative results within 15 min (Fig. 2). The developed *Campylobacter* FIC assay showed 100% detection of *C. jejuni* (**n** = 25), *C. coli* (**n** = 25) and *C. lari* (**n** = 5), but no other bacterial strains (**n** = 56) except for one *C. upsaliensis* strain were detected even when high numbers (6.40-6.70 log CFU) of bacterial cells were applied (Table 1).

**Fig. 2.** Representative images of the *Campylobacter* FIC assay for the detection of *C. jejuni* NCTC 11168. The images were captured by a hand-type scope.

**Table 1.** Specificity of the *Campylobacter* FIC assay.

Bacteria*		No. strains tested	No. positive
Genus *Campylobacter*	*C. jejuni*	25	25
	*C. coli*	25	25
	*C. lari*	5	5
	*C. fetus*	5	0
	*C. upsaliensis*	3	1
	*C. hyointestinalis*	3	0
Other genus	*Escherichia coli*	10	0
	*Salmonella* spp.	10	0
	*Arcobacter butzleri*	10	0
	*Enterobacter* spp.	4	0
	*Klebsiella aerogenes*	1	0
	*Shigella flexneri*	1	0
	*Pseudomonas* spp.	5	0
	*Helicobacter pylori*	5	0

* Bacterial strains tested are as follows: *C. jejuni* NCTC 11168, 81-176, ATCC 33560 and chicken-originating strains (**n **= 22); *C. coli* JCM 2529 and chicken-originating strains (**n **= 24); *C. lari* ATCC 35221, ATCC 35223, ATCC 43675 and chicken-originating laboratory strains (**n **= 2); *C. fetus* ATCC 27374, ATCC 33561 and bovine-originating laboratory strains (**n **= 3); *C. upsaliensis* ATCC 43954, ATCC 49815, ATCC 49816; *C. hyointestinalis* ATCC 35217 and pig-originating laboratory strains (**n **= 2); *E. coli* EDL933, RIMD 0509952(Sakai), Obi-1, WHO1, HP1001, and chicken-originating laboratory strains (**n **= 5); *Salmonella* spp. ATCC 13076, ATCC 53648, ATCC BAA-2568, NCTC 12416 and chicken-originating strains (**n **= 6); *A.butzleri* ATCC 49616, ATCC 49942 and chicken-originating laboratory strains (**n **= 8); *Enterobacter* spp. NBRC 13535, NBRC 109912, NBRC 105718, NBRC 107138; Klebsiella aerogenes NBRC 13534; *Shigella flexneri* YSH6000; *Pseudomonas* spp. NBRC 13275, NBRC 3080, NBRC 14160, NBRC 14164, NBRC 12691; *H. pylori* P12, G27, ATCC 26695, J99, B38.

Recently, immunochromatographic tests, which produce a result within a few minutes and exhibit operational simplicity, have been developed. The first evaluations of these tests showed good sensitivity but an apparent lack of specificity in comparison to those of culture^25^^,^^26^^)^. Given these data, we next examined the sensitivity of the *Campylobacter* FIC assay.

### Sensitivity of the *Campylobacter* FIC Assay

Next, the sensitivity of the *Campylobacter* FIC assay was examined by using different numbers of the *C. jejuni* NCTC 11168 and *C. coli* JCM 2529 strains. The FIC assay detected > 3.08 log CFU of *C. jejuni* NCTC 11168 and > 3.84 log CFU of *C. coli* JCM 2529 (Table 2), even when a hand-type fluorescent image scope was used for the detection (Fig. 2). Statistical analysis revealed that the LOD_50%_ for *C. jejuni* NCTC 11168 or *C. coli* JCM 2529 was approximately 3.51 log CFU or 4.34 log CFU per reaction, respectively (Table 2).

**Table 2.** Estimated limit of detection (LOD) of the *Campylobacter* FIC assay against *C. jejuni* NCTC 11168 and *C. coli* JCM 2529.

Target	LOD_50%_ (log CFU/reaction)				LOD_95%_ (log CFU/reaction)		
	Detection limit	LCL*	UCL†		Detection limit	LCL	UCL
*C. jejuni* NCTC 11168	3.51	3.08	3.93		4.15	3.71	4.57
*C. coli* JCM 2529	4.34	3.84	4.85		4.98	4.48	5.49

* LCL; Lower Confidence Limit, †UCL; Upper Confidence Limit.

A recently developed nanoparticle-based piezoelectric immunosensor integrated with a magnetic immunoseparation system could detect 20-30 CFU of *Campylobacter*, but it requires atomic force microscopy^25^^)^, which is seemingly hard to simultaneously apply to a broad range of slaughterhouses. Another study showed quite a sensitive detection tool for *Campylobacter* using PCR and immunochromatography strips, although it required short-term cultivation prior to genetic detection^26^^)^. Comparatively, our evaluated FIC assay requires fewer instruments without cultivation, and a total detection time of less than 30 min, which seems to be advantageous for possible implementation.

Our future practical study at the poultry slaughterhouse clarifies its possible implications for process hygiene at the facility. Perhaps pretreatment of the sample homogenates with centrifugation might allow the concentration of target microorganisms to obtain enough numbers of *Campylobacter* before loading onto the FIC assay, allowing us to qualitative detection of less numbers of *Campylobacter* in the fields. To examine this possibility, the effects of contaminants other than *Campylobacter*, existing on the poultry carcass skin should be considered because of their complexity^27^^)^. Since poultry processing steps, including scalding, defeathering, evisceration, nick removal, and inside and outside (or inside-out) washing, can all contribute to cross-contamination of *Campylobacter* in one way or another^28^^)^, monitoring of the quantitative dynamics of this pathogen throughout whole processes is expected to reveal the bacterial contamination risks, thereby leading to an adequate control approach at poultry slaughter.
